The article "Protective Effect of Glycyrrhizic Acid on Alcoholic Liver Injury in Rats by Modulating Lipid Metabolism" was retracted in 2019. Reason: errors in the results or conclusions.

# Protective Effect of Glycyrrhizic Acid on Alcoholic Liver Injury in Rats by Modulating Lipid Metabolism

**DOI:** 10.3390/molecules23071623

**Published:** 2018-07-04

**Authors:** Xiaowei Huo, Sa Yang, Xiaoke Sun, Xiangbo Meng, Yanyan Zhao

**Affiliations:** Key Laboratory of Pharmaceutical Quality Control of Hebei Province, College of Pharmaceutical Science, Hebei University, Baoding 071002, China; huoxiaoweiforever@163.com (X.H.); mmliu.bio@gmail.com (S.Y.); liuermengmeng@sina.com (X.S.); liuermengmeng@hotmail.com (X.M.)

**Keywords:** 18α-glycyrrhizic acid, 18β-glycyrrhizic acid, optimal compatibility ratio, alcoholic liver disease

## Abstract

Glycyrrhhizic acid (GA), including 18α-glycyrrhizic acid (18α-GA) and 18β-glycyrrhizic acid (18β-GA), is the main active ingredient of licorice. GA is generally considered an effective pharmacological strategy protecting against hepatic disease; however, the optimal compatibility proportion of 18α-GA and 18β-GA against alcoholic liver disease (ALD) and the underlying mechanism are not well established. Hence, this study was designed to explore the optimal compatibility proportion of 18α-GA and 18β-GA against ALD, followed by investigating the underlying mechanisms. SD rats were administered 40% ethanol once a day, accompanied by treatment with different proportions of 18α-GA and 18β-GA for four weeks. Then all rats were anesthetized with chloral hydrate and blood samples were taken from the abdominal aorta for biochemical assay. Livers were also collected and the liver function, lipid profile, ROS production, and mRNA and protein levels of related genes involved in lipid metabolism were assessed. The results showed that 18α-GA and 18β-GA, particularly at a proportion of 4:6, significantly reduced liver damage, lipid accumulation, and oxidative stress in ethanol-induced rats, as indicated by the decreased levels of alanine aminotransferase (ALT) and aminotransferase (AST) in serum, improvement of liver histopathological changes, regulation of total cholesterol (TC), total triglyceride (TG), high-density lipoprotein cholesterol (HDL-C), and low-density lipoprotein cholesterol (LDL-C), and modulation of superoxide dismutase (SOD), glutathione (GSH), and malonaldehyde (MDA). Moreover, the combination treatment with 18α-GA and 18β-GA substantially reduced the mRNA and protein levels of sterol regulatory element-binding protein-1c (SREBP-1c) and acetyl-coal carboxylase (ACC); meanwhile, increased levels of peroxisome proliferators activated receptor-α (PPAR-α) and carnitine palmitoy transferase-1 (CTP-1) in the liver tissues of ethanol-induced rats. In conclusion, our results indicated that the optimal compatibility proportion of 18α-GA and 18β-GA protecting against ALD was 4:6, and the mechanism was associated with the regulation of oxidative stress and lipid metabolism.

## 1. Introduction

Alcoholic liver disease (ALD) remains a leading cause of morbidity and mortality worldwide [1,2]. The cause of ALD is not well established; however, several studies indicate that alcohol-induced hepatotoxicity, oxidative stress, and complex interactions between alcohol metabolism, hepatic cells, and multiple cytokines may be responsible for the progression of ALD [3,4,5]. The spectrum of ALD includes hepatic steatosis, fibrosis, cirrhosis and hepatocellular carcinoma [6], among which hepatic steatosis has been widely recognized to be the earliest and most common response of the liver to either acute or chronic alcohol exposure [7,8]. In this respect, therapeutic approaches improving hepatic steatosis during alcohol exposure may help to block further liver damage [9].

Natural products derived from herbal medicines are attracting considerable attention as alternative treatment options for prevention and treatment of ALD, largely due to their safety, less side effects, and multi-target actions [10,11]. Licorice, the roots and stolons of some *Glycyrrhiza* species, has been widely used for medicinal purposes for thousands of years [12]. It is also used worldwide in food products as a sweetening and flavoring component owing to its sweet taste. Emerging evidence demonstrates that licorice contains many bioactive components, including flavonoids and triterpenoid. Glycyrrhhizic acid (18α- and 18β-, GA) is a triterpenoid derived from *Glycyrrhiza glabra* L. (licorice) root. Previous investigations of the active components in licorice mainly focused on glycyrrhhizic acid and its derivatives, as they were normally thought to be responsible for the hepatoprotective, antioxidant, anticancer, and anti-inflammatory effects of licorice [13,14,15]. We therefore hypothesize that GA may help to protect against ALD. However, the optimal compatibility proportion of 18α-GA and 18β-GA protecting against ALD has not been studied and the molecular mechanism underlying the effect of GA on ALD remains to be elucidated.

The present study was, therefore, designed to investigate the optimal compatibility proportion of 18α-GA and 18β-GA protecting against liver injury induced by ethanol. Here, we studied the effect of different proportions of 18α-GA and 18β-GA on liver function and lipid profile, and further explored the molecular mechanism against ALD. The results showed that 18α-GA and 18β-GA at a proportion of 4:6 exerted the strongest protection against liver injury induced by ethanol. Additional study revealed that the possible mechanism was associated with its prevention on the development of hepatic steatosis by modulating oxidative stress and hepatic lipid accumulation via regulation of sterol regulatory element-binding protein-1c (SREBP-1c), Acetyl-CoA carboxylase (ACC), peroxisome proliferator-activated receptor-α (PPAR-α), and carnitine palmitocyl transferase-1a (CPT-1a).

## 2. Results

### 2.1. Effect of GA on Body Weight, Liver Index, and Fat Index

The chemical structures of 18α-GA and 18β-GA are shown in Figure 1A,B. The body weight, liver index, and fat index are shown in Figure 1C–F. The body weight in group M decreased significantly compared to the normal control group at the end of the fourth week; however, there was no significant difference in body weight between group M and group GA. The liver index and brown adipose tissue (BAT) index in group M increased significantly when compared with the normal control group, indicating sever lipid and fat accumulation in the liver of rats with ethanol treatment. Fortunately, silybin and the combination treatment with 18α-GA and 18β-GA remarkably decreased the liver index in comparison with ethanol monotherapy; meanwhile, the BAT index in groups P, G2, G5, G6, and G7, particularly group G5 (18α-GA:18β-GA = 4:6), decreased markedly compared with ethanol treatment alone in group M. Additionally, there was no significant difference in the white adipose tissue (WAT) index between all groups. These results indicated that 18α-GA combined with 18β-GA, particularly at a proportion of 4:6, could markedly reduce ethanol-induced liver injury.

### 2.2. Effect of GA on ALT, AST, ALP and GGT

The serum levels of alanine aminotransferase (ALT) and aspartate aminotransferase (AST) have been most commonly used as reliable primary indicators for liver injury [16]. To test the effect of GA on ethanol-induced hepatoxicity, the serum levels of ALT, AST, alkaline phosphatase (ALP) and γ-Glutamyl transferase (GGT) were examined. As shown in Figure 2, the levels of ALT, AST, ALP, and GGT were elevated significantly after ethanol administration. In contrast, the combination treatment with 18α-GA and 18β-GA at proportions of 4:6, 2:8, and 10:0 (groups G5, G6, and G7) significantly dropped the serum levels of ALT, AST, ALP, and GGT, indicating the effective of the combination treatment on protecting against ethanol-induced liver injury.

### 2.3. Effect of GA on Lipid Accumulation

To assess the effect of GA on hepatic lipid accumulation induced by ethanol exposure, lipid content in the serum, liver and fecal matter was examined. As shown in Figure 3, administration of ethanol increased the levels of total cholesterol (TC) and total triglyceride (TG) in serum, liver, and fecal matter as compared to the normal control rats, and GA supplementation significantly prevented this increase. The inhibition of TC and TG was more profound in G5 and G6 groups than in other GA groups. Moreover, 18α-GA combined with 18β-GA at proportions of 4:6, 2:8, and 10:0 (groups G5, G6, and G7) markedly restored the decrease of high-density lipoprotein cholesterol (HDL) and the increase of low-density lipoprotein cholesterol (LDL) caused by ethanol administration. These data clearly indicated that 18α-GA combined with 18β-GA was effective at protecting against ethanol-induced lipid accumulation by decreasing the levels of TC and TG and modulating the levels of HDL and LDL.

### 2.4. Effect of GA on Oxidation Stress

The oxidative stress was regulated by an imbalance of oxidants and antioxidants [17]. To evaluate the effect of GA pretreatment on ethanol-induced oxidative stress, activities and levels of superoxide dismutase (SOD), glutathione (GSH), and malonaldehyde (MDA), successfully used as reliable markers of oxidative stress, were examined in serum and liver tissue. As shown in Figure 4, the serum and hepatic SOD and GSH levels were significantly decreased and MDA level was obviously elevated after ethanol administration compared to that of the untreated rats (group N). The combination treatment with 18α-GA and 18β-GA (groups G5, G6) exerted the strongest protective effect on oxidative stress than the other groups as indicated by the significant increase of SOD and GSH and marked decrease of MDA in these two groups. These results indicated that 18α-GA combined with 18β-GA at the ratio of 4:6 and 2:8 effectively ameliorated ethanol-induced liver injury by modulation oxidative stress via suppressing MDA and increasing levels of SOD and GSH.

### 2.5. Histopathological Observations

The protective effect of GA on the hepatic steatosis in response to ethanol administration was examined by hematoxylin and eosin (H&E) and Oil Red O staining. As shown in Figure 5A, ethanol administration resulted in marked enlargement of hepatocytes and fatty degeneration in the liver tissue compared to that of the normal control group (group N). The combination treatment with 18α-GA and 18β-GA effectively prevented hepatic lipid droplet accumulation and enlargement as documented by H&E staining. Also, the Oil Red O staining showed that the livers of ethanol-treated rats exhibited obvious microvesicular steatosis and large hepatic fatty droplets, which was markedly restored by combination treatment with 18α-GA and 18β-GA (Figure 5B). Moreover, 18α-GA and 18β-GA, particularly at a proportion of 4:6, significantly decreased the steatosis score as compared with the model group (Figure 5C). Taken together, the histological analysis, Oil Red O staining, steatosis score, and lipid profile (Figure 3) confirmed that ethanol administration resulted in significant alcoholic hepatic steatosis and that the combination treatment with 18α-GA and 18β-GA significantly reduced the severity of alcoholic hepatic steatosis in the livers of ethanol-treated rats. These data clearly indicated that 18α-GA and 18β-GA, particularly at a proportion of 4:6, could effectively protect against ethanol-induced hepatic steatosis.

### 2.6. Effect of GA on mRNA and Protein Expression Associated with Lipid Metabolism

We next sought to determine possible mechanisms for the observed protection by the combination treatment with 18α-GA and 18β-GA on ethanol-induced liver injury by evaluating the effects of different proportions of 18α-GA and 18β-GA on mRNA and protein levels of SREBP-1c, ACC, PPAR-α, and CPT-1a involved in lipogenesis and lipolysis in liver tissues. Figure 6 and Figure 7 showed that ethanol treatment elevated the mRNA and protein expression levels of SREBP-1c and ACC, and, meanwhile, decreased the mRNA and protein expression levels of PPAR-α and CPT-1a compared to that of the normal control rats. However, the combination treatment with 18α-GA and 18β-GA, especially at a proportion of 4:6 (group 5), significantly reversed the increase of SREBP-1c and ACC and the decrease of PPAR-α and CPT-1a caused by ethanol treatment. These data indicated that the reason for the protective effect of the combination treatment in response to ethanol administration was likely attributed to the regulation of SREBP-1c, ACC, PPAR-α, and CPT-1a in liver tissues.

## 3. Discussion

To the best of our knowledge, no study has previously been reported investigating the optimal compatibility proportion of 18α-GA and 18β-GA against liver injury. Accordingly, the present study mainly focused on investigating the ameliorative effects of 18α-GA and 18β-GA on ethanol-induced liver injury, and further exploring the mechanisms of action. Rats treated with 18α-GA and 18β-GA, especially at a proportion of 4:6, significantly relieved liver injury induced by ethanol, which was associated with its marked inhibition on lipid accumulation and oxidative stress via regulation of SREBP-1c, ACC, PPAR-α, and CPT-1a.

Previous research has studied the hepatoprotective effect of raw licorice extraction [18]. However, the optimal compatibility proportion of 18α-GA and 18β-GA protecting against ALD has not been investigated. Therefore, the present study mainly focused on investigating the optimal compatibility proportion of 18α-GA and 18β-GA against ethanol-induced liver injury. Here, we found that the combination treatment with 18α-GA and 18β-GA at different proportions, particularly at a proportion of 4:6, alleviated ethanol-induced liver injury, as demonstrated by H&E staining and reduced levels of ALT and AST in serum. Hepatic steatosis, defined histologically as the deposition of fat in hepatocytes, is considered an early consequence of excessive alcohol consumption. Hence, control of hepatic steatosis is essential in the treatment of ALD. In the present study, we found that 18α-GA and 18β-GA, particularly at a proportion of 4:6, could substantially alleviate ethanol-induced hepatic steatosis as evidenced by Oil Red O staining and decreased steatosis score.

Multiple mechanisms contribute to alcoholic hepatic steatosis, involving increased hepatic lipogenesis and inhibited hepatic lipolysis [8]. The excessive lipids in the cytoplasmic of the hepatocytes greatly influence cellular function and cause the hepatocytes to become susceptible to hepatotoxins. Besides, hepatic steatosis is reported to be oxidative stress-associated pathophysiological features of ALD. Thus, therapeutic approaches suppressing hepatic lipid accumulation and controlling oxidative stress during ethanol exposure are beneficial for the treatment of ALD. In the present study, our data showed that the rats intake with ethanol exhibited severe liver damage, increased hepatic lipid accumulation, elevated ROS production, and decreased activities of hepatic GSH, SOD and GPx, which was abolished by the combination treatment with 18α-GA and 18β-GA, especially at a proportion of 4:6. Collectively, the combination treatment with 18α-GA and 18β-GA could alleviate ethanol-induced hepatic steatosis by modulating hepatic lipogenesis and lipidolysis, and also by suppressing oxidative stress.

SREBPs, involving in regulation of lipogenesis, is a family of transcription factors that regulate the enzymes responsible for the synthesis of cholesterol, fatty acids, and triglycerides in liver and other tissues [19,20]. Three SREBP isoforms, designated SREBP-1a, SREBP-1c, and SREBP-2, have been identified [21]. In liver, SREBP-1c mainly regulates lipogenic processes by increasing lipogenic gene expression, enhancing fatty acid synthesis, and accelerating triglyceride accumulation. ACC, the downstream gene of SREBP-1c, is the key gene regulating lipogenesis. ACC catalyzes the irreversible carboxylation of acetyl-CoA to produce malonyl-CoA, which is the rate-limiting step in fatty acid synthesis [20,22]. Ethanol stimulates hepatic fat accumulation by up-regulating SREBP-1c and ACC. Consistently, our study showed that a marked increase of SREBP-1c and ACC could be observed in ethanol-induced rats; however, the combination treatment with 18α-GA and 18β-GA significantly decreased the levels of SREBP-1c and ACC. These findings suggested an effective inhibition of the combination treatment on lipid synthesis via reducing the expression of SREBP-1c and ACC.

PPARs, also involving in lipid metabolism, belongs to nuclear receptor superfamily that controls the expression of genes involved in lipid metabolism, energy homeostasis, and inflammation [23,24]. The PPAR family consists of PPAR-α, PPAR-β, and three isoforms of PPAR-γ [25], among which PPAR-α exists mainly in liver where it controls transcription of genes involved in free fatty acid transport and oxidation [26]. CPT-1a, residing in the outer mitochondrial membrane, is responsive to PPAR-α activation and is a site for the intracellular regulation of lipid metabolism and transporting long-chain fatty acids into mitochondria for β-oxidation, which is widely distributed in the liver, kidneys, brain, pancreas, and embryonic tissues [27,28,29]. Ethanol inhibits the transcriptional activation and DNA binding ability of the PPAR, and its response to ligands [30], thus enhancing fatty acid and triglyceride accumulation. In the present study, our results by RT-PCR and Western blot demonstrated that the combination treatment with 18α-GA and 18β-GA markedly increased levels of PPAR-α and CPT-1a in the liver, indicating the inductive effect of the combination treatment on lipid lypolysis via regulating levels of PPAR-α and CPT-1a. However, other PPARα-targeted genes have not been investigated and the effect of the combination treatment with 18α-GA and 18β-GA on the activity of CPT-1a requires further study.

In summary, our study, for the first time, demonstrated that the optimal compatibility proportion of 18α-GA and 18β-GA against ethanol-induced liver injury was 4:6. The hepatoprotective effect of combination treatment with 18α-GA and 18β-GA in ethanol-treated rats was associated with its strong modulation of oxidative stress and regulation of lipid metabolism via enhancing the expression of PPAR-α and CTP-1; meanwhile, decreasing levels of SREBP-1c and ACC in the liver, as illustrated in Figure 8, through other molecular mechanisms cannot be excluded. 18α-GA and 18β-GA at a proportion of 4:6 may be an effective therapeutic agent to prevent ALD caused by ethanol administration.

## 4. Materials and Methods

### 4.1. Materials and Reagents

Assay kits for ALT, AST, ALP, GGT, TC, TG, HDL-C, LDL-C, SOD, GSH, and MDA were obtained from Nanjing Jiancheng Bioengineering Institute (Nanjing, China). H&E and Oil Red O were purchased from Beijing Solarbio Science & Technology Co., Ltd. (Beijing, China). The TIANScrip RT Kit and Quant qPCR kit were purchased from TIANGEN Biotech (Beijing) Co., Ltd. (Beijing, China). Antibodies (Rabbit) against SREBP-1c (bs-1402R), CTP-1 (bs-2047R), and ACC (bs-2745R) were provided by Beijing Biosynthesis Biothchnology Co., Ltd. (Beijing, China). Antibodies against PPAR-α (ab8934) and horseradish peroxidase (HRP)-conjugated secondary antibodies (ab97051) were purchased from Abcam (Cambridge, UK).

### 4.2. Animal Treatments

Six-week-old male SD rats were purchased from the Sibeifu Laboratory Animal Technology (Beijing, China). All animal experiments were carried out in according to Guide for the Care and Use of Laboratory Animals and the experimental procedures approved by the Animal Care and Ethics Committee at Hebei University. The rats were housed under standard conditions of temperature and humidity with free access to food and water, and were subjected to a 12 h light/dark cycle. After one week of acclimatization, the rats were randomly divided into 10 groups (*n* = 8): (N) normal group, (M) ethanol group, (P) ethanol + silybin group, (G1) ethanol + GA group (18α-GA:18β-GA = 10:0), (G2) ethanol + GA group (18α-GA:18β-GA = 8:2), (G3) ethanol + GA group (18α-GA:18β-GA = 6:4), (G4) ethanol + GA group(18α-GA:18β-GA = 5:5), (G5) ethanol + GA group (18α-GA:18β-GA = 4:6), (G6) ethanol + GA group(18α-GA:18β-GA = 2:8), (G7) ethanol + GA group (18α-GA:18β-GA = 0:10). Rats were orally administrated 40% ethanol and GA for four consecutive weeks. At the end of the fourth week, all rats were fasted for 12 h and anesthetized with chloral hydrate. Blood samples were taken from the abdominal aorta and serum samples were obtained by centrifuging the blood at 3000 rpm for 15 min at 4 °C. Liver, kidney, spleen, and adipose tissues were collected on ice, rinsed with ice-cold physiological saline, and weighed. All tissue samples were snap-frozen in lipid nitrogen and stored at −80 °C for further study.

### 4.3. Biochemical Analysis

Serum ALT, AST, ALP, GGT, TC, TG, HDL-C, LDL-C, TBA, and CHE levels were measured using automatic biochemistry analyzer. Serum SOD, MDA, and GSH levels were measured using commercially available kits following the manufacturer’s instructions. Briefly, livers were homogenized in nine volumes of ice-cold normal saline. The homogenate was extracted with 2 mL chloroform/methanol (2:1, *v*/*v*) for measurement of TC, TG, HDL-C, and LDL-C levels. Additionally, the homogenate was centrifuged at 3000 rpm for 10 min and the supermatant was collected for the measurement of SOD, MDA and GSH.

### 4.4. Hematoxylin & Eosin (H & E) and Oil-Red O Staining

Liver tissues were fixed in 10% neutral buffered formaldehyde or frozen in liquid nitrogen and stored at −80 °C. The fixed livers were cut into 4-µm sections and stained with hematoxylin and eosin for examination of liver histology. Moreover, the frozen livers were cut into 10-µm sections and stained with Oil-Red O and hematoxylin. The sections were then examined by a pathologist blinded to the experimental groups and images of the sections were captured (magnification 100×).

### 4.5. Real Time RT-PCR

Total RNA was extracted from the liver tissue using a TRIzol reagent. The concentration of mRNA was tested by a biophotometer. Total mRNA was converted to first strand cDNA following the instructions provided by the TIANScrip RT Kit. Real-time PCR was performed using a Quant qPCR kit and with a CFX System (Bio-Rad, Hercules, CA, USA). The result was analyzed by the method 2^−△△*C*t^. The primers for RT-qPCR were as follows: SREBP-1c (F: CTATGGAGGGCATGAA, R: AAGGGGCTACTCTGGA); ACC (F: GTGATGGTCTACATTCCCC, R: TACTGTCCCTTCTGGTTCC); PPAR-α (F: AAGAACCTGAGGAAGCCA, R: AGCCACAAAAAGGGAAATG); CTP-1α (F: ACGAAGCCCTCAAACAGA, R: GGATGAAATCACACCCAC); β-actin (F: CTTGCATCCCTCAGCACCTT, R: TCCTGTGGACAATGGATGGA).

### 4.6. Western Blot Analysis

RIPA buffer supplemented with a cocktail of protease and phosphatase inhibitors was used to lyse the liver. Liver protein concentrations of the extracts were measured by a BCA kit according to the manufacturer’s protocol. The proteins were loaded onto 10–15% SDS-PAGE, transferred to polyvinylidene difluoride membranes (PVDF) and blocked with 5% nonfat milk for 1 h. The membranes were incubated overnight with primary antibodies at 4 °C, followed by incubation with horseradish peroxidase (HRP)-conjugated secondary antibodies, then visualized with a chemiluminescence reagent. The protein levels were quantified by the Quantity One Image Analyzer software program (Bio-Rad) and β-actin content was used as an internal control.

### 4.7. Statistical Analysis

The statistical analysis was determined by one-way analysis of variance (ANOVA) followed by Tukey’s post hoc tests. Differences were considered significant when *p* < 0.05. All data are expressed as mean + standard deviation (SD).

## Figures and Tables

**Figure 1:** The chemical structure of 18α-GA (**A**) and 18β-GA (**B**); The effect of GA on body weight (**C**); liver index (**D**); WAT index (**E**); and BAT index (**F**). N: normal group, M: model group, P: silybin positive group, G1: 18α-GA:18β-GA = 10:0, G2: 18α-GA:18β-GA = 8:2, G3: 18α-GA:18β-GA = 6:4, G4: 18α-GA:18β-GA = 5:5, G5: 18α-GA:18β-GA = 4:6, G6: 18α-GA:18β-GA = 2:8, G7: 18α-GA:18β-GA = 0:10. Organ indexes were calculated by the following formula: Organ index = organs weight (g)/body weight (g) × 100%. The values were expressed as mean ± SD (*n* = 8); * *p* < 0.05, ** *p* < 0.01 vs. normal group, ^#^ *p* < 0.05, ^##^ *p* < 0.01 vs. model group.

**Figure 2:** Effect of GA on levels of ALT (**A**); AST (**B**); ALP (**C**); and GGT (**D**) in ethanol-induced rats. N: normal group, M: model group, P: silybin positive group, G1: 18α-GA:18β-GA = 10:0, G2: 18α-GA:18β-GA = 8:2, G3: 18α-GA:18β-GA = 6:4, G4: 18α-GA:18β-GA = 5:5, G5: 18α-GA:18β-GA = 4:6, G6: 18α-GA:18β-GA = 2:8, G7: 18α-GA:18β-GA = 0:10. The values were expressed as mean ± SD (*n* = 8). ** *p* < 0.01 vs. normal group, ^#^ *p* < 0.05, ^##^ *p* < 0.01 vs. model group.

**Figure 3:** The effect of GA on lipid profile, including Serum TC (**A**); Serum TG (**B**); Serum HDL (**C**); Serum LDL (**D**); Liver TC (**E**); Liver TG (**F**); Liver HDL (**G**); Liver LDL (**H**); Fecal TC (**I**); Fecal TG (**J**). N: normal group, M: model group, P: silybin positive group, G1: 18α-GA:18β-GA = 10:0, G2: 18α-GA:18β-GA = 8:2, G3: 18α-GA:18β-GA = 6:4, G4: 18α-GA:18β-GA = 5:5, G5: 18α-GA:18β-GA = 4:6, G6: 18α-GA:18β-GA = 2:8, G7: 18α-GA:18β-GA = 0:10. The values were expressed as mean ± SD (*n* = 8). * *p* < 0.05, ** *p* < 0.01 vs. normal group, ^#^ *p* < 0.05, ^##^ *p* < 0.01 vs. model group.

**Figure 4:** The effect of GA on oxidative stress. Levels of Serum SOD (**A**); Serum MDA (**B**); Serum GSH (**C**); Liver SOD (**D**); Liver MDA (**E**); and Liver GSH (**F**) were determined after GA treatment. N: normal group, M: model group, P: silybin positive group, G1: 18α-GA:18β-GA = 10:0, G2: 18α-GA:18β-GA = 8:2, G3: 18α-GA:18β-GA = 6:4, G4: 18α-GA:18β-GA = 5:5, G5: 18α-GA:18β-GA = 4:6, G6: 18α-GA:18β-GA = 2:8, G7: 18α-GA:18β-GA = 0:10. The values were expressed as mean ± SD (*n* = 8). * *p* < 0.05, ** *p* < 0.01 vs. normal group, ^#^ *p* < 0.05, ^##^ *p* < 0.01 vs. model group.

**Figure 5:** Effect of GA on hepatic histology determined by H&E staining (**A**) and Oil red O staining (magnification 100×) (**B**); Steatosis score (**C**) was graded on a scale of 0 (<5%), 1 (5–33%), 2 (34–66%), and 3 (>66%). N: normal group, M: model group, P: silybin positive group, G1: 18α-GA:18β-GA = 10:0, G2: 18α-GA:18β-GA = 8:2, G3: 18α-GA:18β-GA = 6:4, G4: 18α-GA:18β-GA = 5:5, G5: 18α-GA:18β-GA = 4:6, G6: 18α-GA:18β-GA = 2:8, G7: 18α-GA:18β-GA = 0:10. The values were expressed as mean ± SD (*n* = 8). ** *p* < 0.01 vs. normal group, ^#^ *p* < 0.05, ^##^ *p* < 0.01 vs. model group.

**Figure 6:** Hepatic mRNA expression of SREBP-1c (**A**); ACC (**B**); PPAR-α (**C**) and CPT-1a (**D**) in ALD rats. N: normal group, M: model group, P: silybin positive group, G1: 18α-GA:18β-GA = 10:0, G2: 18α-GA:18β-GA = 8:2, G3: 18α-GA:18β-GA = 6:4, G4: 18α-GA:18β-GA = 5:5, G5: 18α-GA:18β-GA = 4:6, G6: 18α-GA:18β-GA = 2:8, G7: 18α-GA:18β-GA = 0:10. The values were expressed as mean ± SD. ** *p* < 0.01 vs. normal group, ^#^ *p* < 0.05, ^##^ *p* < 0.01 vs. model group.

**Figure 7:** Hepatic protein expression of SREBP-1c, ACC, PPAR-α and CPT-1a in ALD rats. (**A**) Western blot of SREBP-1c, ACC, PPAR-α and CPT-1a and (**B**–**E**) semi-quantitative analysis of these proteins. N: normal group, M: model group, P: silybin positive group, G1: 18α-GA:18β-GA = 10:0, G2: 18α-GA:18β-GA = 8:2, G3: 18α-GA:18β-GA = 6:4, G4: 18α-GA:18β-GA = 5:5, G5: 18α-GA:18β-GA = 4:6, G6: 18α-GA:18β-GA = 2:8, G7: 18α-GA:18β-GA = 0:10. The values were expressed as mean ± SD. ** *p* < 0.01 vs. normal group, ^#^ *p* < 0.05, ^##^ *p* < 0.01 vs. model group.

**Figure 8:** The possible mechanism of GA against ALD.
